The article "Diagnostic Predictive Value of Tryptase, Serum Amyloid A and Lipoprotein-Associated Phospholipase A2 Biomarker Groups for Large Atherosclerotic Cerebral Infarction" was retracted in 2023. Reasons: signs of a paper mill; compromised peer review; unreliable results or conclusions.

# Diagnostic Predictive Value of Tryptase, Serum Amyloid A and Lipoprotein-Associated Phospholipase A2 Biomarker Groups for Large Atherosclerotic Cerebral Infarction

**DOI:** 10.1155/2022/5784909

**Published:** 2022-10-03

**Authors:** Wenhui Jia, Xia Li, Fang Lei, Fengyun Hu, Fenglian Li, Xueying Zhang, Siyu Liu, Feifei Huang, Changxin Li

**Affiliations:** ^1^The Fifth Clinical Medical College of Shanxi Medical University, Department of Neurology, Shanxi Provincial People's Hospital, Taiyuan 030000, China; ^2^Dalian Medical University, Dalian 116000, China; ^3^College of Information and Computer,, Taiyuan University of Technology, Jinzhong 030600, China; ^4^The First Clinical Medical College of Shanxi Medical University, Department of Neurology, Taiyuan 030000, China

## Abstract

**Background:**

There has been a gradual trend towards younger ageing of acute cerebral infarction in recent years. Atherosclerotic plaque rupture followed by dislodgement of emboli and resulting arterial embolism is an important mechanism for the development of acute cerebral infarction. Traditional independent risk factors for cerebral infarction have received attention from clinicians, but the risk factors for large artery atherosclerotic cerebral infarction are still unclear. Various blood biomarkers have an important role in the early diagnosis of large artery atherosclerotic cerebral infarction.

**Objective:**

To assess the diagnostic predictive value of a group of biomarkers for large artery atherosclerotic cerebral infarction.

**Methods:**

Lipoprotein-associated phospholipase A2 (LP-PLA2), trypsin-like protein (TPS), serum amyloid A (SAA), and supersensitive C-reactive protein (hs-CRP) levels were measured in the case group (30 cases) and control group (54 cases), respectively.

**Results:**

The differences in the general data between the two groups were not statistically significant (*P* > 0.05). Logistic regression and ROC curve analysis showed that Lp-PLA2, TPS, and SAA were positively associated with the diagnosis of large atherosclerotic cerebral infarction (*P* < 0.05). The area under the ROC curve of the multivariate model for the biomarker group reached 0.995.

**Conclusion:**

Biomarkers are closely associated with the occurrence of large atherosclerotic cerebral infarction and can be used as clinical adjuncts for diagnosis and assessment of prognosis.

## 1. Introduction

Stroke has a high recurrence, disability, and mortality rate, and places a heavy economic and psychological burden on society and the patient's family. Ischemic strokes account for approximately 80% of all strokes. The treatment of ischemic strokes is not limited to symptomatic treatment (salvage of ischemic brain tissue), but also to the diagnosis and treatment of the cause, which has been unanimously accepted by neurologists [1]. The diagnosis of ischemic stroke based on TOAST etiological staging [2], followed by treatment planning and recurrence prevention, plays an important role in the management of stroke. With the widespread use of TOAST etiology in clinical practice, the incidence of LAAS in each subtype has been found to be increasing in recent years. A study by Chen et al. [3] found that the incidence of LAAS accounted for 16.5% of patients in the Yonsei Stroke Registry in Korea when examining the risk factors and subtypes of 1000 patients with acute cerebral infarction. The study by Dobrocky et al. [4] found that LAAS accounted for 25.3% of all TOAST subtypes, second only to cardiogenic embolism (46.2%); the study by Zhou et al. [5] found that small artery occlusion and LAAS were the most common (44.2% and 37.6%, respectively) when reporting the relationship between acute cerebral infarction TOAST staging and risk factors. Although the results of domestic and international studies vary, the prevalence of LAAS among TOAST subtypes is relatively high in China. Because patients with LAAS have severe intracranial and extracranial large artery stenosis or occlusion, the potential for disability, death, and recurrence of stroke remains high with aggressive pharmacological and nonpharmacological interventions, and should therefore be studied with emphasis [6].

At present, the diagnosis of acute cerebral infarction (ACI) relies mainly on imaging, but many primary care institutions lack equipment such as head MRI and CT and do not have the capacity to complete relevant examinations in a timely manner. In contrast, early identification, etiological typing, disease assessment, risk stratification, and prognostic assessment of ACI, as well as personalised treatment plans, are of great clinical and social importance. In cardiology and respiratory emergency cases, such as troponin for acute myocardial infarction and D-dimer for early diagnosis of pulmonary embolism are of great value [7]. We lack a widely used, rapid, and sensitive blood biomarker for the clinical diagnosis of ACI, so finding a blood biomarker that can rapidly diagnose ACI is a clinical imperative. However, not much research has been done in this area.

Previous studies have shown that the levels of several blood biomarkers (ultrasensitive C-reactive protein, lipoprotein-associated phospholipase A2, and metalloproteinase-9) are elevated to varying degrees during the acute phase of ischemic stroke, but changes in a single marker have limitations for the diagnosis of ischemic stroke [8, 9]. Therefore, we screened four indicators widely reported in the literature, hs-CRP, TPS, Lp-PLA2, and SAA, all of which have been shown in several studies to be atherosclerotic inflammatory factors [10, 11].

Based on this, 84 patients with large atherosclerotic cerebral infarction were selected for this study, and the levels of TPS, Lp-PLA2, SAA, and hs-CRP were measured in patients with LAA, and the diagnostic predictive value of the four biomarkers for LAA was further evaluated to provide the reference value for clinical application.

## 2. Materials and Methods

### 2.1. General Information

Select 100 consecutive cases of acute cerebral infarction diagnosed in the Department of Neurology of Shanxi Provincial People's Hospital from January 2021 to January 2022, of which 30 inpatients with large atherosclerotic cerebral infarction (LAA) by TOAST etiology typing were selected, including 20 males and 10 females with an average age of (62.37 ± 14.11) years, and another age-sex matched fifty-four cases were selected as the control group with age- and sex-matched healthy physical examiners.

### 2.2. Diagnostic Criteria

All cases of cerebral infarction met the diagnostic criteria for cerebral infarction established by the Chinese guidelines for the diagnosis and treatment of acute ischemic stroke 2018 [12], were confirmed by cranial magnetic resonance imaging (MRI); patients with first-onset cerebral infarction were hospitalized within 72 hours of onset, and the 100 patients with acute cerebral infarction enrolled were classified as large atherosclerotic cerebral infarction according to the TOAST etiological typing in the Org 10172 trial of acute stroke treatment.

### 2.3. Inclusion and Exclusion Criteria

All met the following inclusion criteria: (1) the diagnostic criteria established by the 4th National Cerebrovascular Disease Conference [13] and confirmed by cranial CT/MRI; (2) could cooperate with the completion of routine blood and serum biomarker tests; (3) gave informed consent to the study and voluntarily signed the informed consent form. The exclusion criteria include the following: (1) those who are unable to complete serum biomarker tests; (2) those with major organ diseases such as heart, liver, or kidney; (3) those with previous cerebral haemorrhage, subarachnoid haemorrhage, traumatic brain injury, or haematological disorders; (4) those with a clear history of tuberculosis, syphilis, connective tissue disease, or other diseases that can cause vascular damage; (5) those who are unable to cooperate with the completion of this study.

### 2.4. Experimental Method

General information including gender, age, previous medical history (hypertension, hyperlipidaemia, and, diabetes), smoking and alcohol consumption was recorded. Blood specimens were collected on the morning of the second day of admission and biomarkers were measured. High-sensitivity C-reactive protein (hs-CRP) was measured by reflectance turbidimetry, brain natriuretic peptide (BNP) by immunofluorescence, and fibrinogen (FIB) by immunoturbidimetry, all measured on a Beckman coulter AU5800 fully automated biochemistry analyser. Lipoprotein-associated phospholipase A2 (Lp-PLA2), myelin basic protein (MBP), and glial fibrillary acidic protein (GFAP) were measured by ELISA, the kits were purchased from eBioscience, and the enzyme standard was a GO full wavelength enzyme standard from Thermo Fisher, USA. Normal reference values were as follows: hs-CRP 0.1–10 mg/L, BNP 0–38 pg/ml, FIB 2–4 g/L, Lp-PLA2 ≤ 175 ng/ml, MBP ≤ 80 ng/L, and GFAP ≤ 1.0 ng/L.

### 2.5. Statistical Methods

All data were statistically analysed using SPSS 22.0 software, measures were expressed as mean ± standard deviation (*x* ± *s*), the *t*-test was used for the measurement data and the *χ*^2^-test was used for the count data, binomial classification logistic regression was used to screen the variables and establish the regression equation to generate a new set of variables. ROC curve analysis was performed for the new variables and each individual index, and *P* < 0.05 was considered statistically different.

## 3. Results

### 3.1. Comparison of General Clinical Information between the Case Group and the Control Group

The differences in gender, age, smoking history, drinking history, and BMI between the case group and the control group were not statistically significant (*P* > 0.05), indicating an equal distribution of general information between the two groups (Table 1).

### 3.2. Comparison of Lipids, Fasting Glucose, Uric Acid, and White Blood Cell Count between the Case Group and the Control Group

The differences in CHO, HDL-C, LDL, UA, and blood WBC levels between the case group and the control group were not statistically significant (*P* > 0.05), and the differences in TG and fasting glucose levels were statistically significant (*P* < 0.05) (Table 2).

### 3.3. Comparison of Biomarkers between Case and Control Groups

The levels of serum hs-CRP, LP-PLA2, SAA, and TPS in the case group were significantly higher than those in the control group, and the differences were statistically significant by the *t*-test (*P* < 0.05). HCY and FIB were not statistically significant between the two groups (*P* > 0.05) (Table 3).

### 3.4. Logistic Regression Analysis of the Three Biomarkers

Logistic regression analysis showed that among the three biomarkers, TPS, Lp-PLA2, and SAA were positively correlated with the diagnosis of the acute phase of atherosclerotic cerebral infarction (*P* < 0.05), while the correlation of hs-CRP was not significant (*P* > 0.05) (Table 4).

### 3.5. ROC Curve Analysis of the Diagnostic Value of Three Biomarkers Alone and in Combination for the Acute Phase of Atherosclerotic Cerebral Infarction

Logistic regression analysis in this study showed that the area under the curve (AUC) of the three biomarkers was TPS > SAA > Lp-PLA2 with a maximum value of 0.935, and SAA was positively correlated with the acute phase diagnosis of LAA (*P* < 0.05) with an area under the curve (AUC) of 0.916, suggesting a high clinical value for ACI diagnosis and prediction (Table 5 and Figure 1).

## 4. Discussion

A widely used, rapid and sensitive diagnostic test is still lacking in the acute phase of ischemic stroke. In some other medical emergencies, diagnostic tests based on blood biomarkers have become a routine. For example, troponin, creatine kinase, brain natriuretic peptide, and D-dimer play an important role in the early diagnosis of acute myocardial infarction, heart failure, and pulmonary embolism. Previous studies have shown that the levels of several blood biological markers (ultrasensitive C-reactive protein, lipoprotein-associated phospholipase A2, and metalloproteinase-9) are increased to varying degrees during the acute phase of ischemic stroke [14], but changes in a single marker have limitations for the diagnosis of ischemic stroke. In China, atherosclerotic cerebral infarction is an important subtype of TOAST etiology, so in this study, six blood biomarkers associated with atherosclerotic cerebral infarction were screened to form a biomarker panel (lipoprotein-associated phospholipase A2 (Lp-PLA2) A2 (Lp-PLA2), myeloperoxidase (MPO), matrix metalloproteinase-9 (MMP-9), myeloperoxidase (MPO), matrix metalloproteinase-9 (MMP-9), hypersensitive C-reactive protein (Hs-CRP), fibrinogen (FIB), and brain natriuretic peptide (BNP)). Logistic regression analysis and ROC curves were used to investigate the diagnostic value of biomarker groups in the acute phase of atherosclerotic cerebral infarction.

LP-PLA2 is a novel inflammatory marker that has been extensively studied both nationally and internationally as a key enzyme mediating the inflammatory effects of ox-LDL and promoting AS formation [15]. The Rotterdam study [16] (Rotterdam Study and TRS Study), a prospective case-cohort study, confirmed for the first time that serum Lp-PLA2 is a new independent predictor of cerebral infarction. Numerous domestic and international studies have shown that LP-PLA2 is closely associated with AS and cerebral infarction, is a risk factor for ACI, predicts the prognosis of ACI, and is a predictor of ACI recurrence [17]. A study by Luo et al. [18] found that elevated Lp-PLA2 levels in patients with atherosclerotic cerebral infarction were positively correlated with NIHSS scores, which has an important clinical value for the diagnosis and treatment of atherosclerotic cerebral infarction. Related studies have further shown that Lp-PLA2 is closely associated with large vessel stenosis and may even serve as a potential biomarker for predicting the degree of cerebrovascular stenosis in patients with ACI [19]. The results of this study showed that serum LP-PLA2 levels were significantly higher in LAA patients than in controls and were positively correlated with the diagnosis of the acute phase of LAA. ROC curve analysis showed that the area under the curve was 0.822, indicating that LP-PLA2 was closely associated with the occurrence of LAA and had diagnostic predictive value for the acute phase of LAA.

The study by Kang et al. [20] reported for the first time that it is synthesized by hepatocytes, secreted and involved in the formation and development of AS, promoting the formation of AS plaques, leading to plaque rupture and thrombosis. The study by Lee et al. [21] confirmed that SAA accelerates atherosclerotic plaque progression in apolipoprotein *E* knockout mice. In recent years, several domestic and international studies have shown that SAA can initiate and develop atherosclerosis through a series of proinflammatory and proatherogenic activities that have been clearly shown to influence the progression of atherosclerosis and may be a candidate target for clinical trials in cardiovascular disease [22]. SAA is not only a marker of cardiovascular disease but also an early atherosclerotic process participant [23]. The study by Leng et al. [24] concluded that SAA is a useful biomarker for the diagnosis of atherosclerotic thrombotic ischemic stroke. In addition, several studies confirmed that SAA is one of the most sensitive markers of inflammation in the acute phase of cerebral infarction [25]. Several foreign studies have concluded that SAA levels can assess the severity of acute cerebral infarction and determine the prognosis [26]. The study by Sun et al. [27] found that SAA levels were significantly and positively correlated with ACI and were a risk factor for ACI. Logistic regression analysis in this study showed that SAA was positively correlated with the diagnosis of acute phase of LAA (*P* < 0.05) with an area under the curve (AUC) of 0.916, suggesting a high clinical value for ACI diagnosis and prediction.

TPS is a natural protease with multiple biological activities that may be involved in the development and progression of AS by preventing reverse HDL cholesterol transport, aggregating inflammatory cells, and other mechanisms leading to atherosclerotic plaque formation and rupture. In recent years, the relationship between TPS and AS has been increasingly studied, with TPS emerging as a new inflammatory marker for AS. The study by Tsang et al. [28] concluded that TPS levels significantly correlated with carotid intima-media thickness were higher in patients with carotid plaque and independently predicted changes in subclinical atherosclerosis. An experimental study in monkeys and hamsters found that TPS inhibition blocked macrophage foam cell formation and reduced atherosclerotic plaque formation [29]. It was found [30] that TPS inhibited LXR*α* activation through the PAR-2/LXR*α*/LXR*α* target gene signaling pathway, which promoted macrophage lipid accumulation and foam cell formation, further promoting AS formation. However, there are few studies on the correlation between TPS and large atherosclerotic cerebral infarction, and the present study found that after studying LAA patients and normal controls, TPS levels in the case group were significantly different from those in the control group, and logistic regression analysis showed that TPS was positively correlated with the diagnosis of acute phase of LAA, and TPS was further associated with LAA, with an area under the curve (AUC) of 0.935, suggesting that the diagnosis and prediction of ACI has a high clinical value.

In this study, the inflammatory markers LP-PLA2, SAA, and TPS associated with LAA were selected, and the levels of each inflammatory marker were found to be elevated during the acute phase of cerebral infarction. Logistic regression analysis showed that LP-PLA2, SAA, and TPS were positively correlated with LAA (*P* < 0.05), and all were independent risk factors for LAA. Analysis of these three biomarkers used to diagnose LAA using ROC curves showed that TPS had the highest AUC value of 0.935 if a single indicator was used to diagnose LAA. A new variable *Y* was generated by multiple logistic regression analysis combining the three biomarkers, and the area under the ROC curve used to diagnose the new variable *Y* was obtained by plotting the ROC curve at 0.995 and the value of the new variable *Y* was higher than the area of any individual indicator. It can be seen that by detecting the TPS biomarker set, SAA and Lp-PLA2 are more valuable than one alone, increasing the specificity and sensitivity of LAA diagnosis to more than 99%, which is valuable for rapid diagnosis and pathogen typing of LAA.

## 5. Conclusions

The results of this study suggest that the combined detection of multiple biomarkers is an effective means to improve the clinical value of ischemic stroke diagnostic tests. It is although the complexity of the stroke process and the specificity of the brain tissue structure, the sensitivity and specificity of stroke biomarkers have been the main problems faced by stroke biomarker research. However, we found that TPS, Lp-PLA2, and SAA were significantly higher, and the area under the ROC curve of the multivariate model LP-PLA2, SAA, and TPS combined reached 0.995. The sensitivity and specificity of the combined prediction group for the diagnosis of LAA was extremely high, which has a high clinical value for the diagnosis of LAA and can provide a reference value for clinical application, and is worthy of further promotion in our clinical practice.

## Figures and Tables

**Figure 1:** ROC curves for the new variable *Y* and the three biomarkers.

**Table 1:** Comparison of general clinical information between the case and control groups.

−	−	Case group	Control group	*χ* ^2^	*P*
Gender	Male	20	36	0.0	1.0
	Female	10	18		
Smoking	Yes	16	19	2.613	0.106
	No	14	35		
Drinking	Yes	9	12	0.622	0.430
−	No	21	42		
*−*	*−*	*Number of cases*	$\bar{x}\pm s$	*t*	*P*
Age	Case group	30	62.37±14.11	1.952	0.054
−	Control group	54	55.96±14.57	−	−
BMI	Case group	30	24.86±2.28	0.731	0.467
−	Control group	54	24.40±3.40	−	−

**Table 2:** Comparison of blood lipids, fasting glucose, uric acid, and white blood cell count between the case group and the control group.

-	−	Number of cases	$\bar{x}\pm s$	*t*	*P*
CHO	Case group	30	4.24±1.15	0.609	0.544
(mmol/L)	Control group	54	4.39±1.01	−	−
TG	Case group	30	1.27±0.46	2.37	0.02
(mmol/L)	Control group	54	1.63±0.93	−	−
HDL-C	Case group	30	1.13±0.45	1.379	0.172
(mmol/L)	Control group	54	1.29±0.54	−	−
LDL	Case group	30	2.78±0.91	0.678	0.5
(mmol/L)	Control group	54	2.65±0.81	−	−
Blood sugar	Case group	30	6.06±1.97	3.149	0.002
(mmol/L)	Control group	54	5.07±0.84	−	−
UA	Case group	30	285.91±68.08	0.151	0.881
(*μ*mol/L)	Control group	54	288.83±91.36	−	−
WBC	Case group	30	6.84±1.86	1.759	0.086
(×10^9^/L)	Control group	54	6.07±1.88	−	−

**Table 3:** Comparison of each biomarker index between the case group and the control group.

−	−	Number of cases	$\bar{x}\pm s$	*t*	*P*
Hs-CRP	Case group	30	8.81±10.82	3.503	0.001
(mg/L)	Control group	54	2.37±5.04	−	−
LP-PLA_2_	Case group	30	396.60±233.34	3.191	0.003
(ng/L)	Control group	54	251.94±110.71	−	−
SAA	Case group	30	1589.23±788.28	6.389	<0.001
(ng/L)	Control group	54	646.78±231.32	−	−
TPS	Case group	30	11.80±6.37	6.848	<0.001
(ng/ml)	Control group	54	3.81±0.73	−	−
HCY	Case group	30	26.93±18.11	0.986	0.331
(*μ*mol/L)	Control group	54	21.79±11.77	−	−
FIB	Case group	30	3.23±0.61	0.243	0.809
(g/L)	Control group	54	3.26±0.49	−	−

**Table 4:** Logistic regression analysis of large artery atherosclerotic cerebral infarction.

Biomarkers	Regression coefficient	Standard error	OR	*P*
Constants	−26.811	11.798	0.000	0.023
TPS	1.441	0.680	4.226	0.034
SAA	0.012	0.006	1.012	0.045
LP-PLA2	0.023	0.012	1.023	0.045

**Table 5:** AUC of single biomarker and combined assay for predicting probability of new variable *Y*.

Test items	AUC	Standard error	*P*	95%CI	
				Lower limit	Upper limit
TPS	0.935	0.037	<0.001	0.863	1.000
SAA	0.916	0.037	<0.001	0.843	0.988
Lp-PLA2	0.822	0.046	<0.001	0.731	0.912
*Y*	0.995	0.004	<0.001	0.987	1.000

*Y*-value = TPS + SAA + Lp-PLA2.

## Data Availability

The experimental data used to support the findings of this study are available from the corresponding author upon request.

## References

[1] Zhang H., Zhao X., Wang C. (2019). A preliminary study of the association between apolipoprotein E promoter methylation and atherosclerotic cerebral infarction. *Journal of Stroke and Cerebrovascular Diseases*.

[2] Li Q., Liu M., Fu R. (2018). Alteration of circulating innate lymphoid cells in patients with atherosclerotic cerebral infarction. *American Journal of Tourism Research*.

[3] Chen L., Yang Q., Ding R., Liu D., Chen Z. (2018). Carotid thickness and atherosclerotic plaque stability, serum inflammation, serum MMP-2 and MMP-9 were associated with acute cerebral infarction. *Experimental and Therapeutic Medicine*.

[4] Dobrocky T., Kaesmacher J., Bellwald S. (2019). Stent-retriever thrombectomy and rescue treatment of M1 occlusions due to underlying intracranial atherosclerotic stenosis: cohort analysis and review of the literature. *Cardiovascular and Interventional Radiology*.

[5] Zhou D., Li J., Liu D. (2019). Irregular surface of carotid atherosclerotic plaque is associated with ischemic stroke: a magnetic resonance imaging study. *Journal of Geriatric Cardiology: JGC*.

[6] Ni T., Fu Y., Zhou W. (2020). Carotid plaques and neurological impairment in patients with acute cerebral infarction. *PLoS One*.

[7] Wang Y., Xu S., Pan S., Ouyang H., Zang Z., Tan J. (2018). Association of serum neuron‐specific enolase and bilirubin levels with cerebral dysfunction and prognosis in large‐artery atherosclerotic strokes. *Journal of Cellular Biochemistry*.

[8] Yan Z., Fu B., He D., Zhang Y., Liu J., Zhang X. (2018). The relationship between oxidized low-density lipoprotein and related ratio and acute cerebral infarction. *Medicine*.

[9] Anniwaer J., Liu M. Z., Xue K. D., Maimaiti A., Xiamixiding A. (2019). Homocysteine might increase the risk of recurrence in patients presenting with primary cerebral infarction. *International Journal of Neuroscience*.

[10] Wu L., Qian L., Zhang L. (2020). Fibroblast growth factor 21 is related to atherosclerosis independent of nonalcoholic fatty liver disease and predicts atherosclerotic cardiovascular events. *Journal of American Heart Association*.

[11] Wang G. J., Dong X., Li Y. (2022). Cluster of Differentiation 147 (CD147) serves as a promoter of atherosclerosis in patients with cerebral infarction. *European Review for Medical and Pharmacological Sciences*.

[12] Kang D. H., Yoon W., Kim S. K. (2019). Endovascular treatment for emergent large vessel occlusion due to severe intracranial atherosclerotic stenosis. *Journal of Neurosurgery*.

[13] Kim H., Kim S., Han S. (2019). Prevalence and incidence of atherosclerotic cardiovascular disease and its risk factors in Korea: a nationwide population-based study. *BMC Public Health*.

[14] Zhang W. B., Zeng Y. Y., Wang F., Cheng L., Tang W. J., Wang X. Q. (2020). A high neutrophil-to-lymphocyte ratio predicts hemorrhagic transformation of large atherosclerotic infarction in patients with acute ischemic stroke. *Aging (Albany NY)*.

[15] Ouchi Y., Sasaki J., Arai H. (2019). Ezetimibe lipid-lowering trial on prevention of atherosclerotic cardiovascular disease in 75 or older (ewtopia 75) A randomized, controlled trial. *Circulation*.

[16] Yang D., Lin M., Wang S. (2018). Primary angioplasty and stenting may be superior to thrombectomy for acute atherosclerotic large-artery occlusion. *Interventional Neuroradiology*.

[17] Hassan A. E., Ringheanu V. M., Preston L., Tekle W. G., Qureshi A. I. (2022). Acute intracranial stenting with mechanical thrombectomy is safe and efficacious in patients diagnosed with underlying intracranial atherosclerotic disease. *Interventional Neuroradiology*.

[18] Luo J., Wang T., Gao P., Krings T., Jiao L. (2018). Endovascular treatment of intracranial atherosclerotic stenosis: current debates and future prospects. *Frontiers in Neurology*.

[19] Feng X., Chan K. L., Lan L. (2019). Stroke mechanisms in symptomatic intracranial atherosclerotic disease: classification and clinical implications. *Stroke*.

[20] Kang D. H., Yoon W. (2019). Current opinion on endovascular therapy for emergent large vessel occlusion due to underlying intracranial atherosclerotic stenosis. *Korean Journal of Radiology*.

[21] Lee H. N., Ryu C. W., Yun S. J. (2018). Vessel-wall magnetic resonance imaging of intracranial atherosclerotic plaque and ischemic stroke: a systematic review and meta-analysis. *Frontiers in Neurology*.

[22] Gross B. A., Desai S. M., Walker G., Jankowitz B. T., Jadhav A., Jovin T. G. (2019). Balloon-mounted stents for acute intracranial large vessel occlusion secondary to presumed atherosclerotic disease: evolution in an era of supple intermediate catheters. *Journal of Neurointerventional Surgery*.

[23] Liu Y. U., Cheng J., Guo X. (2018). The roles of PAI-1 gene polymorphisms in atherosclerotic diseases: a systematic review and meta-analysis involving 149, 908 subjects. *Gene*.

[24] Leng X., Lan L., Ip H. L. (2019). Hemodynamics and stroke risk in intracranial atherosclerotic disease. *Annals of Neurology*.

[25] Liu Y., Wang M., Zhang B. (2019). Size of carotid artery intraplaque hemorrhage and acute ischemic stroke: a cardiovascular magnetic resonance Chinese atherosclerosis risk evaluation study. *Journal of Cardiovascular Magnetic Resonance*.

[26] Ghuman M., Tsang A. C. O., Klostranec J. M., Krings T. (2019). Sentinel angiographic signs of cerebral hyperperfusion after angioplasty and stenting of intracranial atherosclerotic stenosis: a technical note. *AJNR. American journal of neuroradiology*.

[27] Sun R., Wang L., Guan C., Cao W., Tian B. (2018). Carotid atherosclerotic plaque features in patients with acute ischemic stroke. *World Neurosurgery*.

[28] Tsang A. C. O., Orru E., Klostranec J. M. (2019). Thrombectomy outcomes of intracranial atherosclerosis-related occlusions: a systematic review and meta-analysis. *Stroke*.

[29] Hoshino T., Sissani L., Labreuche J. (2018). Prevalence of systemic atherosclerosis burdens and overlapping stroke etiologies and their associations with long-term vascular prognosis in stroke with intracranial atherosclerotic disease. *JAMA Neurology*.

[30] Xu W., Xie N., Zhang C., Huang Q. (2018). Imaging characteristics and pathogenesis of intracranial artery stenosis in patients with acute cerebral infarction. *Experimental and Therapeutic Medicine*.

